The article "Study of cell apoptosis in the hippocampus and thalamencephalon in a ventricular fluid impact model" was published in 2013. Journal: Exp Ther Med.

# Study of cell apoptosis in the hippocampus and thalamencephalon in a ventricular fluid impact model

**DOI:** 10.3892/etm.2013.1342

**Published:** 2013-10-11

**Authors:** RUI CHEN, JUNYU WANG, BING JIANG, XIN WAN, HONGWEI LIU, HUAN LIU, XIAOSHENG YANG, XIAOBING WU, QIN ZOU, WENREN YANG

**Affiliations:** 1 Department of Neurosurgery, Xiangya Hospital of Central South University, Changsha, Hunan 410008, P.R. China; 2 Department of Cardiology, Nanhua Hospital Affiliated to Nanhua University, Hengyang, Hunan 421001, P.R. China; 3 Department of Neurosurgery, Nanhua Hospital Affiliated to Nanhua University, Hengyang, Hunan 421001, P.R. China

**Keywords:** ventricular fluid, hippocampus, thalamencephalon, apoptosis, pathological change

## Abstract

The aim of this study was to investigate the apoptosis of nerve cells in the hippocampal and thalamencephalon regions using a rabbit model of ventricular fluid impact. The results for the study demonstrated a variety of pathophysiological changes in the rabbit model, while changes in the hippocampal and thalamencephalon regions were observed under a light microscope following hematoxylin and eosin (H&E)/terminal deoxynucleotidyl transferase dUTP nick end labeling (TUNEL) staining. Among the mild, moderate and severe injury groups, there were significant differences in the mortality rate and in the changes in vital signs and consciousness recovery time following trauma. Furthermore, H&E staining showed that pathological changes, such as hemorrhage and necrosis, occurred in the hippocampal and thalamencephalon regions at an early stage subsequent to trauma, while TUNEL staining showed that neuronal apoptosis occurred in the various injury groups. In traumatic brain injuries, the impact caused by cerebrospinal fluid moving with a certain energy results in marked damage to the contralateral periventricular structures and may generate a series of pathophysiological changes.

## Introduction

Common traumatic brain injury models are mainly divided into two types: the impact injury and the acceleration injury models (1–3). The impact injury model is achieved by keeping the animal in a stationary state and drilling a window into the skull. Focal and diffuse brain injuries may be generated by the impact of a liquid or the steel body of the drill on the dura mater, resulting in damage to the brain tissue via the bone window. The model demonstrates good experimental control and reproducibility. The acceleration injury model (3) is further subdivided into two models: simple inertial acceleration and acceleration impact injuries. The former entails fixing the animal in a controllable acceleration device and causing a linear or rotational acceleration motion injury, according to the design requirements, rather than by directly impacting the brain. The significant feature of this model is that it enables independent investigation of the inertia damage mechanism. The acceleration impact injury is characterized by the traditional Feeney’s falling body method (4). In this model, the head of the animal is kept stationary and a heavy object is dropped from a high position to impact and damage the head. The main features of the acceleration impact injury model include the fact that it is possible to adjust the extent of the injury by altering the height that the object falls from and the weight of the object. Furthermore, it is easy and simple to repeat the acceleration brain injury.

The article "Study of cell apoptosis in the hippocampus and thalamencephalon in a ventricular fluid impact model" was published in 2013. Journal: Exp Ther Med.

However, these animal models only consider brain injuries caused by the transmission of external forces to the brain, and ignore the fact that brain is composed of multiple tissues rather than being one homogeneous body. The mechanical properties of the tissues comprising the brain are inconsistent and there is a certain volume of cerebrospinal fluid in the brain ventricles. The cerebrospinal fluid and the surrounding brain tissue are two different types of substance. Furthermore, the cerebrospinal fluid is incompressible (5,6). In the deceleration injury process, the brain tissue impacts the skull over a short stretch of time, while the cerebrospinal fluid impacts the ventricular wall more slowly. The impact caused by the cerebrospinal fluid moving with a certain energy results in injuries to the periventricular structures.

Cell apoptosis may be observed in various traumatic brain injury models, and studies have suggested that cell apoptosis is involved in the whole process of secondary pathophysiological evolution following craniocerebral injury (7,8). However, to the best of our knowledge, there have not been any studies investigating whether cerebrospinal fluid moving with a certain energy causes injuries to periventricular structures, resulting in cell apoptosis in the deceleration injury process. Therefore, the authors designed a ventricular fluid impact model, in order to simulate the situation of the cerebrospinal fluid impacting the ventricular wall during the deceleration injury process. The aim of this was to observe the changes in various indicators of the animal at different levels of energy and to investigate the occurrence of apoptosis of the nerve cells in the periventricular structures, the hippocampus and thalamencephalon.

## Materials and methods

### Grouping

A total of 88 New Zealand rabbits with a mean body weight of 2.5±0.3 kg (provided by the Experimental Zoology Department of Central South University, Changsha, China) were randomly divided into normal control, surgical control and injury groups. For the former two groups, each group comprised eight rabbits, whereas the injury group comprised 72 rabbits. According to the principle of randomization, the injury group was further divided into the following three subgroups: mild, moderate and severe injury (24 rabbits in each subgroup). Eight rabbits were randomly selected from each injury group to determine consciousness recovery time following trauma (in the mild, moderate and severe injury groups there were eight, seven and three survival cases used, respectively, to determine the consciousness recovery time following trauma). Variations in respiration, blood pressure and heart rate were monitored. In each group, the remaining 16 rabbits, respectively, were used for pathological examinations following brain perfusion fixation conducted at 12 h and 1, 2, 3 and 7 days subsequent to trauma (in the mild, moderate and severe injury groups, there were 15, 13 and 10 survival cases, respectively, used for the determination of the apoptosis-positive cell count). This study was carried out in strict accordance with the recommendations in the 8th Edition of the Guide for the Care and Use of Laboratory Animals (January 1, 2012). The animal use protocol was reviewed and approved by the Institutional Animal Care and Use Committee (IACUC) of Xiangya Hospital of Central South University.

The article "Study of cell apoptosis in the hippocampus and thalamencephalon in a ventricular fluid impact model" was published in 2013. Journal: Exp Ther Med.

### Device used for animal brain injury

The device used for the animal brain injury consisted of five components: a weight, a free falling body device (reference to Feeney’s method), a 5-ml syringe (adequately lubricated), a ventricular drainage tube and a holder. The lower part of the free falling body device was connected to the syringe, while the lower part of the syringe was connected to the lateral ventricle through the ventricular drainage tube. The top part of the weight was fixed with a threadlet onto the upper part of the device. The threadlet length was adjusted. As the weight dropped to impact the upper syringe core and move it down by 0.8 cm (~1.0 ml liquid flowed out from the syringe), the threadlet over the weight was tightened, and the weight did not drop again. Therefore, the liquid entered the lateral ventricle through the ventricular drainage tube. Immediately subsequent to this, the holder was moved away (Fig. 1).

### Surgical technique and experimental procedure

Nembutal solution (30 g/l) was slowly injected at a dose of 33 mg/kg via an intravenous injection to the marginal ear vein. Following successful anaesthesia, a rabbit was fixed onto the holder in prone position and, under aseptic conditions, the sutura was exposed. In accordance with the method by Kockro *et al*(9), a small hole with a diameter of 1.5 mm was drilled by a dental drill on the right side of 4 mm of the middle line at the crown drill joint, prior to the venous indwelling needle (outer diameter of 1.1 mm, replacing the lateral ventricular drainage tube) being inserted by 4–6 mm. Following the removal of the internal core, the cerebrospinal fluid rose in the silicone tube, indicating the success of the puncture, and it was fixed with dental resin. The right femoral artery catheter was connected to a blood pressure monitor and the femoral vein catheter was connected to the infusion set. Heart rate and respiration were monitored by a physiological recorder. A weight of 100 g fell from heights of 23, 53 and 94 cm for the mild, moderate and severe injury groups, respectively, to impact the upper syringe core (according to the energy conservation law mgh=½mv^2^, the converted impact energy was equivalent to the energy generated by 15 ml cerebrospinal fluid in a human unilateral ventricle momentarily impacting the ventricle wall at speeds of 20, 30 and 40 km/h, respectively, prior to slowing and stopping). Subsequently, the holder was immediately moved away and the ventricular drainage tube was removed. An injection of gentamycin sulfate (40,000 U) was dripped onto the incision for 4–5 days, prior to the bone window being sealed with bone wax and the scalp being sutured. For the surgical control group, only the lateral ventricle puncture was conducted, without the impact procedure. For the normal control group, no intervention was conducted.

The article "Study of cell apoptosis in the hippocampus and thalamencephalon in a ventricular fluid impact model" was published in 2013. Journal: Exp Ther Med.

### Specimen acquisition

The groups of animals were conventionally anaesthetized, respectively, at the preset time-points. Following perfusion fixation with 4% paraformaldehyde, brain tissues were extracted, conventionally dehydrated, hyalinized and embedded with paraffin wax for hematoxylin and eosin (H&E) and immunohistochemical staining.

### Analysis of results

Cell apoptosis was evaluated with the cell apoptosis detection kit provided by Boster Biotecimology Ltd., Co. (Wuhan, China) according to the terminal deoxynucleotidyl transferase dUTP nick end labeling (TUNEL) method. If brown granules were present in the cell nucleus, the cell was positive for apoptosis. In combination with positive H&E staining results, where cells that were positive for apoptosis displayed circular and shrinkage morphology characteristics, cells with nuclear pyknosis, deep cell staining and structural integrity were considered to be apoptotic nerve cells. Under the light microscope, five fields of view were randomly selected to conduct the cell count. The mean positive cell count of 100 cells was calculated and taken as the apoptosis index (10).

The article "Study of cell apoptosis in the hippocampus and thalamencephalon in a ventricular fluid impact model" was published in 2013. Journal: Exp Ther Med.

### Statistical analysis

All data are expressed as the mean ± standard deviation. For a comparison of the same indicator at different time-points, a t-test was used. One-way analysis of variance (ANOVA) was used for comparisons of data from different injury groups, and a non-parameter Kruskal-Wallis test was used to evaluate inter-group heterogeneity of variance. SPSS 13.0 statistical software (SPSS, Inc., Chicago, IL, USA) was used for statistical processing. P<0.05 was considered to indicate a statistically significant difference.

## Results

### Pathophysiological changes

The mortality rates for the mild, moderate and severe injury groups were 4.16, 16.67 and 45.83%, respectively. There were significant differences between the three groups (P<0.05). The time of death of all cases was within 1 h subsequent to trauma, and there were no deaths in the normal or surgical control groups.

In contrast to the normal and surgical control groups, the mild and moderate injury groups immediately presented with exaggerated and deep respiration following trauma, while the severe injury group immediately presented with apnea. Subsequent to the respirator being connected, the majority of the surviving animals regained autonomous respiration within 10–15 min following the trauma. Compared with the normal and surgical control groups, the differences at 2 h subsequent to trauma were not significant.

All the traumatized animals immediately demonstrated an elevation in mean arterial pressure following the trauma, with the pressure reaching a peak at 5 sec subsequent to the trauma. The animals then presented with hypopiesia for some time. Within 15–30 min, the mean arterial pressure returned to the level prior to trauma, whereas the blood pressure of the fatally injured animals continually dropped until death.

The mean heart rate of the animals that survived following trauma rapidly decreased from 238±39 beats/min to 160±61 beats/min and gradually returned to the level prior to trauma within 15–30 min. By contrast, the mean heart rate of the fatally injured animals decreased to 50% of the level prior to trauma in 2 min and then continually declined until death.

The corneal reflex was normal in the normal control and the surgical control groups. In the case of acupuncture, the animals presented evasive actions and were able to crawl by themselves. It was indicated that consciousness returned to the normal level (11) (Table I).

### Pathological changes

Examinations of the normal control and surgical control groups under a light microscope were normal. H&E staining of the hippocampus showed that the morphological structures of the hippocampus in the mild injury group were normal at various time-points subsequent to trauma. By contrast, the morphological structures of the hippocampus in the moderate injury group at 24 h subsequent to trauma underwent significant changes; the tissues were loose and hemorrhagic foci were visible. Similar results were observed in the severe injury group at 8 h subsequent to trauma (Fig. 2A), i.e. the morphological structures of the hippocampus were significantly changed; however, the changes were more marked than those of the moderate injury group. H&E staining of the thalamencephalon showed that the morphological structures of the thalamencephalon in the mild injury group were normal at various time-points subsequent to trauma, although slight intercellular edema was present at 24 h. The cellular structures of the moderate injury group at 24 h were extensively changed; intercellular edema was present and few or no hemorrhagic foci were visible; by contrast, the changes in the cellular structures of the severe injury group at 8 h were more evident, nuclear pyknosis was visible and there was marked intercellular edema (Fig. 2B).

The article "Study of cell apoptosis in the hippocampus and thalamencephalon in a ventricular fluid impact model" was published in 2013. Journal: Exp Ther Med.

TUNEL staining showed that very few cells were positive for apoptosis in the normal control and surgical control groups. With regard to the injury groups, TUNEL staining of the hippocampus showed that there was a small number of cells positive for apoptosis in the mild injury group at 48 h subsequent to trauma and the peak number was reached at 72 h subsequent to trauma. In the moderate and severe injury groups, apoptotic cells were present at 24 h subsequent to trauma and the peak number was reached at 72 h (Fig. 3). At 7 days subsequent to trauma, levels of apoptotic cells had dropped markedly (Table II).

The trend revealed by the TUNEL staining of the thalamencephalon was consistent with that of the hippocampal staining. In the mild injury group a small number of apoptotic cells were present at 48 h subsequent to trauma, and the number peaked at 72 h subsequent to trauma. Apoptotic cells were observed in the moderate and severe injury groups at 24 h, with the number peaking at 72 h (Fig. 4) and markedly declining at 7 days (Table III).

## Discussion

The majority of common traumatic brain injury animal models only consider brain injuries caused by the transmission of external forces to the brain (12–14); however, these models ignore the fact that the brain is composed of multiple tissues rather than being one homogeneous substance. The mechanical properties of these tissues differ and there is a certain volume of cerebrospinal fluid in the brain ventricles. The cerebrospinal fluid and the surrounding brain tissue are two different types of substance (15,16). Furthermore, the cerebrospinal fluid is incompressible. In the deceleration injury process, the brain tissue impacts the skull over a short stretch of time, while the cerebrospinal fluid impacts the ventricular wall more slowly. The impact caused by the cerebrospinal fluid moving with a certain energy results in injuries to the periventricular structures. In this study, based on the previously mentioned considerations, the mathematical principle was closely combined with the physical principle and a free falling body device was used to generate a constant and reproducible graded energy by energy conservation law calculation, and the energy was transmitted to the brain ventricle via a ventricular drainage tube to simulate the situation of the cerebrospinal fluid impacting the ventricular wall during the deceleration injury process. The aim of this was to observe the changes in various vital indicators of the animal at different levels of energy and to investigate the occurrence of nerve cell apoptosis in periventricular structures, specifically, in the hippocampus and thalamencephalon.

The article "Study of cell apoptosis in the hippocampus and thalamencephalon in a ventricular fluid impact model" was published in 2013. Journal: Exp Ther Med.

In the current study, TUNEL positive cell determination in the hippocampus revealed that injury extent was correlated with the time of the occurrence of cell apoptosis; the earlier the occurrence of apoptosis, the greater the number of apoptotic cells. This suggests that, within a certain energy range, the greater the energy of the ventricle trauma, the more severe the extent of hippocampal injury and the greater the number of hippocampal cells positive for TUNEL staining are likely to be. If the energy exceeded the energy limit, it is likely to induce the necrosis of a number of cells. Light microscopy and electron microscopy studies have demonstrated that, in the case of cerebral concussion, the cerebral cortex and hippocampus show diffuse neuronal morphological changes (13,17). This model indicated that simple ventricular fluid impact induced neuronal cell apoptosis in the hippocampus constituting the wall of the ventricular temporal horn. This type of pathological change is likely to be one of the anatomical bases for cerebral concussion presenting with dysmnesia. In addition, functional disorder manifestations of the respiratory cycle of the animals in this model were similar to the transient brainstem responses following cerebral concussion. It is possible that, in the case of deceleration injury, the impact of intraventricular cerebrospinal fluid on periventricular structures is just a complementary explanation among cerebral concussion pathogeneses.

The article "Study of cell apoptosis in the hippocampus and thalamencephalon in a ventricular fluid impact model" was published in 2013. Journal: Exp Ther Med.

Previous studies have suggested that persistent ischemia and degeneration in the thalamencephalon following trauma may be important in severe brain trauma, particularly in the case of animal survival (12,18,19), since the thalamencephalon is located at the sides of the three ventricles and the lateral ventricle. In the current study, the possible impact of ventricular liquid on the lateral ventricle during deceleration injury was considered, and it was demonstrated using the TUNEL immunohistochemical staining method that cell apoptosis was persistent in the thalamencephalon. In this model, there was no significant difference in the animal consciousness recovery time between the mild injury and the control groups. The animal consciousness recovery time of the moderate and severe injury groups were significantly extended compared with those of the control group, with the mean animal consciousness recovery time of the severe injury group reaching 7.83±4.0 h. However, cell apoptosis in the thalamencephalon occurred relatively early, at 24 h subsequent to trauma. Therefore, extension of the animal consciousness recovery time in this study was not observed to correlate with the levels of cell apoptosis. H&E staining showed that the moderate and severe injury groups presented with hemorrhagic necrotic changes in the thalamencephalon at 2 h subsequent to trauma. This suggests that the extension in animal consciousness recovery time at this time was due to cell necrosis rather than cell apoptosis in the acute stage of trauma. In the case of secondary brain injury, the main form of cellular death becomes apoptosis. This long-term phenomenon of cell apoptosis in the thalamencephalon, as a result of ventricular liquid impact, may be one of the important reasons for persistent coma in patients with craniocerebral trauma subsequent to trauma injury.

In conclusion, nerve cell apoptosis was apparent in the ventricular fluid impact model, and the reason for the apoptosis was closely associated with the impact of the ventricular liquid on the periventricular structures. The results of this study may be beneficial in the further development of new understandings of the pathological mechanism of clinical craniocerebral injury and its pathological changes (20–23).

## Figures and Tables

**Figure 1:** The weight was fixed with a threadlet. When the weight dropped, the threadlet was tightened and the liquid in the syringe flowed into the ventricle.

**Figure 2:** Hematoxylin and eosin staining of the (A) hippocampus (nuclear pyknosis was visible and intercellular substance presented obvious edemas, as shown by the black arrow head) and (B) thalamencephalon in the severe injury group at 8 h subsequent to trauma (magnification, ×100).

The article "Study of cell apoptosis in the hippocampus and thalamencephalon in a ventricular fluid impact model" was published in 2013. Journal: Exp Ther Med.

**Figure 3:** Terminal deoxynucleotidyl transferase dUTP nick end labeling (TUNEL) staining of sections of the hippocampus in the moderate injury group at (A) 24 h and (B) 3 days subsequent to trauma (magnification, ×100).

**Figure 4:** Terminal deoxynucleotidyl transferase dUTP nick end labeling (TUNEL) staining of sections of the thalamencephalon in the severe injury group at (A) 3 and (B) 7 days subsequent to trauma (magnification, ×400).

**Table I:** Consciousness recovery time of rabbits following brain injury.

Group	n	Consciousness recovery time (h)
Normal control	8	2.00±0.39
Surgical control	8	2.11±0.40
Mild injury	8	2.43±1.20
Moderate injury	7	5.85±1.23
Severe injury	3	7.83±0.40

Data are presented as the mean ± standard deviation. For comparisons between the normal control group and the surgical control and mild injury groups, the P-values were 0.672 and 0.364, respectively, and there were no significant differences (P>0.05). For comparisons between the normal control group and the moderate and severe injury groups, the P-values were 0.034 and 0.013, respectively, and there were significant differences (P<0.05). For a comparison between the moderate injury and severe injury groups, the P-value was 0.027 and the difference was significant (P<0.05).

**Table II:** Comparison of the apoptosis index in the hippocampal CA1 region of rabbits following trauma.

		Time after trauma				
		
Group	n	12 h	1 day	2 days	3 days	7 days
Normal control	8	1.03±1.32	-	-	-	-
Surgical control	8	1.01±0.90	-	-	-	-
Mild injury	15	1.21±1.21	1.13±0.27	8.19±2.13	12.18±1.96	7.56±2.74
Moderate injury	13	1.97±0.88	6.21±2.37	12.15±2.19	18.44±3.97^a^	8.93±2.51
Severe injury	10	1.13±1.12	8.23±1.81	15.35±3.11	27.18±5.05^b^	9.12±3.04

Significant differences (P<0.05) were identified in the cell apoptosis index at 3 days subsequent to trauma between ^a^the moderate injury group and the mild injury group (P=0.035) and ^b^the severe injury group and the moderate injury group (P=0.042).

**Table III:** Comparisons of the apoptosis index in the thalamencephalon of rabbits following trauma.

		Time subsequent to trauma				
		
Group	n	12 h	1 day	2 days	3 days	7 days
Normal control	8	1.72±0.86	-	-	-	-
Surgical control	8	1.84±0.73	-	-	-	-
Mild injury	8	1.89±0.82	1.88±0.87	16.38±5.92	27.29±8.93	13.92±4.21
Moderate injury	8	1.91±0.76	17.45±6.73	19.68±8.81	34.25±6.25^a^	12.88±3.27
Severe injury	8	1.80±0.72	20.17±8.84	29.11±9.60	43.47±10.29^b^	13.15±6.78

Significant differences (P<0.01) were identified in the cell apoptosis index at 3 days subsequent to trauma between ^a^the moderate injury group and the mild injury groups (P=0.008) and ^b^the severe injury group and the moderate injury groups (P=0.023).
